# Experimental Analysis of Fabricated Synthetic Midthoracic Paediatric Spine as Compared to the Porcine Spine Based on Range of Motion (ROM)

**DOI:** 10.1155/2021/2799415

**Published:** 2021-09-24

**Authors:** Nor Amalina Muhayudin, Khairul Salleh Basaruddin, Ruslizam Daud, Fiona McEvoy, Tansey

**Affiliations:** ^1^Faculty of Mechanical Engineering Technology, Universiti Malaysia Perlis, 02600, Pauh Putra Campus, Perlis, Malaysia; ^2^Faculty of Electronic Engineering Technology, Universiti Malaysia Perlis, 02600 Perlis, Malaysia; ^3^Sports Engineering Research Centre, Centre of Excellence (SERC), Universiti Malaysia Perlis, 02600 Perlis, Malaysia; ^4^Mechanical Engineering Department, Institute of Technology Tallaght, Dublin, Dublin 24, Ireland

## Abstract

The present study is aimed at investigating the mechanical behaviour of fabricated synthetic midthoracic paediatric spine based on range of motion (ROM) as compared to porcine spine as the biological specimen. The main interest was to ensure that the fabricated synthetic model could mimic the biological specimen behaviour. The synthetic paediatric spine was designed as a 200% scaled-up model to fit into the Bionix Servohydraulic spine simulator. Biomechanical tests were conducted to measure the ROM and nonlinearity of sigmoidal curves at six degrees of freedom (DOF) with moments at ±4 Nm before the specimens failed. Results were compared with the porcine spine (biological specimen). The differences found between the lateral bending and axial rotation of synthetic paediatric spine as compared to the porcine spine were 18% and 3%, respectively, but was still within the range. Flexion extension of the synthetic spine is a bit stiff in comparison of porcine spine with 45% different. The ROM curves of the synthetic paediatric spine exhibited nonlinearities for all motions as the measurements of neutral zone (NZ) and elastic zone (EZ) stiffness were below “1.” Therefore, it showed that the proposed synthetic paediatric spine behaved similarly to the biological specimen, particularly on ROM.

## 1. Introduction

Human adult and animal cadaveric spines such as porcine, sheep, baboon, and calf are commonly used in biomechanical investigation [1–5]. Over the years, the understanding of human spinal biomechanics was based on comprehensive studies of human adult spine [1, 3, 5]. On the other hand, information on paediatric spinal biomechanics was very limited due to difficulties in obtaining paediatric human cadavers. Although paediatric and adult spines were distinctively different from each other in both anatomically and mechanically, studies on paediatric spines started by scaling down from the adult size model to paediatric size model in finite element analysis [6–10]. The studies on paediatric spine started with manipulation of the adult finite element model to the paediatric model to incorporate anatomical differences between adult and paediatric spines. Although there were distinct differences between adult and paediatric spines such as the morphology of their vertebra, the orientation of facet joints was more horizontal in the paediatric spine and thus made it more mobile as compared to the adult spine and ossification state of the vertebrae and size of nucleus pulposus were larger in the paediatric intervertebral disc as compared to adult disc. Paediatric spine is not miniature of adult spine; therefore, it cannot be treated as such. A few studies on paediatric biomechanical investigation still used human adult and immature porcine spine as their specimens due to the limitations of paediatric specimens [11–13]

The main challenge in developing the paediatric biomechanical analyses was limited information of paediatric experimental data to enable a direct comparison with the finite element model. Recently, a few studies were reported on the use of paediatric human cadavers to investigate the paediatric biomechanical response [3, 14]. Ouyang et al. [15] investigated bending and tensile tests of paediatric cervical spines from neck to head of 2 years old to 12 years old. The study found that the distraction load for 6 years old to 12 years old was significantly higher as compared to 2 to 4 years old. Another study to investigate the failure tolerance was conducted by Lopez-Valdes et al. [3] by using human paediatric and adult thoracic spines. Similar findings were found by Lopez-Valdes et al. whereby 7-year-old spines showed lower tolerance as compared to 15-year-old spines. The study suggested that the 15-year-old spine tolerance was comparable to adult spines. On the other hand, Clarke et al. [14] used sheep spines to investigate the biomechanical differences between mature and immature spines by using newborn and 2-year-old specimens. The study focused on ROM and found that immature spines (newborn specimens) exhibited a significantly lower ROM as compared to mature spines (2 years old). In paediatric in vivo testing, these were the only studies found as a guide to compare the synthetic paediatric spine with human paediatric spine. This limitation of paediatric human spines can be overcome by developing a working synthetic paediatric spine. Hence, more biomechanical testing in regards with paediatric spines can be performed such as paediatric trauma during motor vehicle collision, paediatric sports-related injuries, and other common recreational injuries that required paediatric specimens for further investigations.

Development of a synthetic paediatric spine is essential to investigate the mechanical behaviour of paediatric cases such as scoliosis. The common surgical procedure among paediatric cases is early onset scoliosis surgical treatment, and studies on the effect and accuracy of various paediatric spinal instrumentations of scoliosis normally were conducted only using FE studies, animal spines, or postoperative studies that required years of observation [11, 16, 17]. Therefore, it will be beneficial to have a working synthetic paediatric spine that can be used in spinal instrumentations of biomechanical investigations or preplanning of complicated surgical treatment. The main advantage in using synthetic materials is that they can be tailored to a specific requirement, and they offer constant material properties. On the hand, studies conducted by Suh et al., Du et al., and Oroszlány et al. [18–20] proved that thoracic was the most common affected region in spine with more than 50% cases amongst children. Therefore, the present study was focused on the synthetic spine development of the thoracic region, particularly on T4-T8. In recent years, synthetic materials were commonly used as alternatives in biomechanical testing, especially in trabecular bone [21–24]. Bohl et al. started to develop adult synthetic spine model of L3-L5 segments by using a 3D printer, and they found that although there were great differences in ROM data, the study claimed that the model could mimic a specific ROM on standard ROM testing applied to cadavers [25, 26]. The present study is mainly aimed at developing a working synthetic paediatric spine as another alternative in paediatric spine biomechanical testing. The key element is to ensure that the synthetic model performs similarly to the biological model. Therefore, the objective of this paper is to investigate the ROM of synthetic midthoracic paediatric spine as compared to porcine spine.

## 2. Methods

The first step in synthetic paediatric spine fabrication was the development of physical paediatric spine model. Since the actual physical size of paediatric model was relatively small to be tested with the MTS Bionix Servohydraulic spine simulator, a scaling process was considered. To the author's knowledge, no data on physiological ROM of human paediatric spine exists, particularly in the thoracic region, and thus, it is essential to generate an experimental protocol by using biological specimens before ROM of the synthetic spine was determined.

### 2.1. Scaling of Paediatric Spine

Another important factor that was considered while developing the synthetic paediatric spine was the actual size of human paediatric spine. Assuming that size of the paediatric spine is 100%, the size of adult spine is normally scaled up to 141%, and the size of porcine spine is larger than an adult spine by an average difference of 50% [4, 27, 28]. Therefore, the porcine spine size is approximately 190% as compared to paediatric spine. In this research, the synthetic paediatric spine was scaled up to 200% of the paediatric spine size to fit the size of the MTS Bionix Servohydraulic system spine simulator which was in reference to the size of porcine spine that was used as the cadaver control data as shown in Figure 1.

A physical model of paediatric vertebra was purchased from Sawbones (Inc., Vashon Island, USA) for all regions, and these vertebrae represent the anatomical dimension of a juvenile group (8 to 9 years old). Since this study focused on T4-T8, five individual vertebrae were scanned in three-dimension (3D) before being scaled to 200% in a selective laser sintering (SLS) machine to fabricate the prototype.

### 2.2. Fabrication of Synthetic Paediatric Spine

The materials to fabricate the synthetic spine were divided into three main components, which were vertebra, intervertebral disc, and spinal ligaments. All materials used in the synthetic paediatric spine were structurally and mechanically close to human data. This was to ensure that the final product (synthetic paediatric spine) could replicate human behaviour. Details of analysis to select the material for each component of spine are available in previous author's publications, namely, for vertebra [4], intervertebral disc [5], and spinal ligament [6].  Table 1 summarises the properties of the selected materials for each component of fabricated synthetic paediatric spine.

The paediatric synthetic spine was fabricated as a single functional spinal unit (FSU), consisting of two vertebrae, an intervertebral disc, and associated ligaments. The process started with embedding the cortical around the trabecular structure. Next, the disc was attached within the two vertebrae by using the “spinous processes” natural structure as reference. The next process was to mould the spinal ligaments within the posterior elements and attach the anterior longitudinal ligament (ALL) and posterior longitudinal ligament (PLL) within the vertebral body. Finally, the vertebral body was covered with sheet wax. All materials used in the synthetic paediatric spine were geometrically and mechanically close to human data. The fabrication process flow is summarised in Figure 2.

### 2.3. Biomechanical Testing

To provide an indication of whether the materials selected to fabricate the synthetic paediatric spine could mimic human spine movement or not, a series of experiments were carried out for both porcine spine and synthetic paediatric spine.

#### 2.3.1. Specimen Preparation

Six porcine spines from 6 months to 7 months old were provided from a local abattoir. The breed was a cross Saddleback with Gloucester porcine. Average weight of spines used was 82.34 kg (±4.9 kg). The full spines were freshly dissected into single FSUs (T4-T5, T5-T6, T6-T7, and T7-T8) with three specimens for each FSU, as shown in Figure 3. All ligaments, disc, and vertebra were preserved, while muscle tissues were carefully removed and frozen at -20°C. The specimens were thawed for 24 hours before testing. The specimens were potted to ensure that the middle disc was aligned horizontally with the spine simulator. The upper half of top vertebra and lower half of bottom vertebra were embedded in a polyurethane liquid plastic (Smooth Cast 300).

Four FSUs of synthetic paediatric spine from T4 to T8 were prepared based on the fabrication process mentioned in Section 2.2, with three specimens for each FSU. All twelve specimens were potted to ensure that the middle disc was aligned horizontally with the spine simulator. Similar to porcine specimens, the upper half of top vertebra and lower half of bottom vertebra were embedded in liquid resin (Smooth Cast 300).

#### 2.3.2. Experimental Setup

These experiments were conducted by using MTS Bionix Servohydraulic system spine simulator. Specimens were fixed at its natural position in the spine simulator before testing, as shown in Figure 4. Twelve specimens were then tested without a preload to avoid buckling in an alternating sequence of flexion/extension, lateral bending right/left, and axial rotation right/left under pure moments. All specimens were tested at five cycles, and the first two cycles were considered as precycles. The applied moments and angular displacements were recorded for each cycle. The experiments were performed under ±7.5 Nm load with 1.7 deg/sec for all DOF, and the results used were at the fifth cycle.

All specimens were tested to obtain flexion, extension, right and left lateral bending, and right and left axial rotation by using the MTS Bionix Servohydraulic spine simulator under similar experimental procedures developed prior to the porcine spine test. To observe the performance of synthetic paediatric spine, three specimens were tested until failure by using a pure moment of ±1 Nm (0.1 deg/sec) for all six DOF with an increment of ±1 Nm. Results from these three specimens showed that the specimens failed at ±5 Nm, whereby the disc started to detach from the vertebrae. Therefore, an assumption was made that the valid ROM for the paediatric synthetic spine in this study was at ±4 Nm. The rest of specimens were tested at ±4 Nm with 1 deg/sec rate. All specimens were tested to five cycles, whereby the first two cycles were considered as the precycle and results were determined at the fifth cycle.

#### 2.3.3. Analysis of ROM

ROM was determined from the sigmoidal curve for each loading direction from the fifth cycle: flexion, extension, right and left lateral bending, and right and left axial rotation. The typical curve for each loading direction is shown in Figure 5. The arrows indicated the loading and unloading direction. Key parameters in the curve are total ROM, NZ ROM, NZ stiffness (S1), and EZ stiffness (S2).

Results collected from synthetic paediatric spine test were plotted in the sigmoidal curve to observe if any nonlinearity existed in the ROM. The nonlinearities or sigmoidal patterns were essential to prove that the synthetic paediatric spine exhibited a viscoelastic behaviour, which is normally found in the biological specimens. The nonlinearities of graphs were observed for all specimens, as it was the key parameter to determine the performance of synthetic spine as compared to the biological specimens. The value of S1/S2 was expected to be lower than 1.0 to prove that the curve was a nonlinear curve, whereby the smaller the value, the stronger the sigmoidicity.

## 3. Results and Discussions

### 3.1. ROM of Porcine Spine

The ROM data for each FSU at ±7.5 Nm moment is summarised in Table 2. The data showed that for flexion extension, T5-T6 and T7-T8 were stiffer than T4-T5 and T6-T7 by around 40%. In lateral bending, all FSUs were in good agreement with less than 10% difference between each FSU. As for axial rotation, difference between the biggest ROM (T6-T7) and lowest ROM (T4-T5) was around 30%. Interestingly, T4-T5 and T6-T7 results came from the same specimens. In this research, specimen 2 was the most flexible porcine spine. Overall, all FSUs showed the same pattern, whereby it increased from flexion extension to lateral bending and axial rotation, except for T4-T5. The wide interspecimen variability was expected as each FSU was from a different porcine spine specimen.

As for ROM at moment of ±4 Nm, it increased from flexion extension to lateral bending and axial rotation, except for T5-T6. The differences between each FSU in each DOF were only around 20%, except for T5-T6. Data indicated that T5-T6 in axial rotation was the stiffest as compared to other FSUs and DOF. The ROM data for each FSU at ±4 Nm moment is summarised in Table 3.

### 3.2. ROM of Synthetic Paediatric Spine

Variables of interest were the ROM and value of S1/S2, as summarised in Table 4. In Table 4, axial rotation exhibited more linear curves as compared to other ROMs because the average value of S1/S2 was 0.7, which was closed to 1.0. The most nonlinear curves were observed in lateral bending with an average value of 0.16. In flexion and extension curves, the upper FSUs (T4-T5 and T5-T6) showed more linear curves as compared to lower FSUs (T6-T7 and T7-T8). Although axial rotation curves were inclined towards a linear curve, the values of S1/S2 for all cases were still lower than 1.0, which suggested that all six DOF exhibited nonlinearity curves in their ROMs.

The second variable was ROM of each FSU, whereby the pattern that emerged for ROM values showed distinct differences between FSUs. The results can be divided into two groups, which were the upper FSUs (T4-T5 and T5-T6) and lower FSUs (T6-T7 and T7-T8) in all six DOF. The upper FSUs and lower FSUs were within the same range for all six DOF. The percentage differences within upper FSUs and lower FSUs were more than 50% for all six DOF. Flexion/extension was the stiffest motion, followed by lateral bending and axial rotation. Despite differences between FSUs, the pattern emerged similar to the pattern showed in porcine spine, whereby the ROM increased from flexion/extension to axial rotation.

## 4. Discussion

The biomechanical analysis of a spine was normally carried on a single FSU. Despite testing a small segment of the spine, it can exhibit the characteristics of the entire spine. Due to limited information on the physiological ROM of paediatric spine, the porcine spine was an essential substitute to guide in biomechanical testing. The physiological ROM included were flexion and extension, left and right lateral bending, and left and right axial rotation. The series of tests were conducted on porcine spines from T4 to T8 on a single FSU under ±7.5 Nm moments at all six DOF. The ROM was measured for all six DOF at ±7.5 Nm moments and was directly compared with a previous study on porcine spines by Wilke et al. [2], since the average weight for tested porcine spines was within the same range used in this research.

In Figure 6, the flexion/extension of the porcine spines presented was varied in all FSUs. The flexion/extension of T4-T5 and T6-T7 was 20% different as compared to research but was within the range. In contrast, T5-T6 and T7-T8 had 50% average difference with that in literature and T7-T8 flexion was the only DOF that was within the range. On the other hand, the average of lateral bending and axial rotation was in good agreement and was within the range obtained by Wilke et al. [2] for all FSUs, as presented in Figure 6.

The average of all FSUs for the midthoracic region (T4-T8) is summarised in Figure 7 in all six DOF. The difference between lateral bending and axial rotation was less than 2%, while flexion/extension was stiffer by 36% [7]. The significant difference in flexion/extension might be potentially due to weight and size of the porcine tested. Although the ROM in lateral bending and axial rotation from these FSUs were within the range provided by literature, the average was lower as compared to other FSUs. As suggested by Muhayudin et al. and White and Panjabi, specimen weight played a significant effect on the anatomical spine dimension, which may subsequently affect the ROM and in this research, whereby it significantly affected the flexion/extension [28, 29]. Therefore, by considering the differences in flexion/extension between current study and literature, the results of porcine spine from this study were used in the comparative analysis with synthetic paediatric spine.

Since no data is available on ROM of human paediatric spine, further analysis was required to compare the porcine ROM with human adult ROM from White and Panjabi under the same moment [29]. The ROM presented in Figure 8 was an average ROM measurement taken from a single FSU, ranging from T4 to T8. As expected, both sets of porcine data were comparable, except for flexion/extension. However, when compared to human adult ROM, the differences ranged from 60% to 90% for all six DOF. In lateral bending and axial rotation, the differences between porcine and human adult ROMs were approximately around 93% and 66%, respectively. In contrast, the flexion/extension from this study was comparable to human adult with 12% difference, while Wilke et al. was 74% larger than that of a human adult. The size of porcine spines was evidently larger than human adult spines, which subsequently resulted in a larger ROM. However, the relation between specimen size and ROM was not linear as the material properties, specifically the viscoelasticity of the soft tissues which was different for each specimen. This was considered when the comparative analysis was conducted between the synthetic paediatric and porcine spine.

The crucial element in testing synthetic paediatric spine was to ensure that the plotted curve showed nonlinearities to replicate the viscoelastic behaviour of soft tissues in human spine. Therefore, the first parameter was to determine the ratio of EZ stiffness (S1) to NZ stiffness (S2). In Table 4, axial rotation exhibited more linear curves as compared to other ROMs because the average value of S1/S2 was 0.7, which was close to 1.0. The most nonlinear curves were observed in lateral bending with an average value of 0.16. In flexion and extension curves, the upper FSUs (T4-T5 and T5-T6) showed more linear curves as compared to lower FSUs (T6-T7 and T7-T8). Although axial rotations curve were inclined towards linear curve, the values of S1/S2 for all cases were still lower than 1.0, which suggested that all six DOF exhibited nonlinearity curves in their ROMs.

The nonlinear behaviour in ROM was a result from both soft and hard tissues. The lateral bending exhibited nonlinear curves with a ratio closer to 0, suggesting that the materials selected as synthetic intervertebral disc replicated the human behaviour. The lateral bending movement was dependent on the nonlinearity of intervertebral disc as the facet joints made less contact with each other. As for the axial rotation and flexion/extension, the nonlinearity curves measured were closer to 1, which suggested that the ROM tended to be more linear. These movements involved facet contacts that tended to be stiffer due to stiffness of the bone. This was potentially caused by assuming that the facet joints had the same material properties as spinal ligaments.

The ROM of porcine was compared to synthetic paediatric spine at ±4 Nm moments. As the size of synthetic paediatric spine (200%) and porcine spine (190%) was 10% different, the average ROM was expected to differ, but was still within the same range. Two assumptions were made in the comparative analysis. The assumptions were that the relation between specimen size and ROM was not linear, and that the synthetic paediatric spine was fabricated by using synthetic material, which did not necessarily exhibit all the behaviour of biological soft tissues. Theoretically, the synthetic materials used in the synthetic paediatric spine were supposed to allow wider movement as compared to the human adult spine. Therefore, the ROM of synthetic paediatric spine was expected to be within the same range as porcine spine, because the porcine ROM was larger than the human adult ROM (Figure 8).

Generally, porcine spine ROM was more flexible as compared to synthetic paediatric spine in all six DOF, with a larger difference in flexion/extension by 45%. The flexion and extension was expected to be lower in the synthetic paediatric spine as compared to the porcine spine because the experimental data of all synthetic paediatric spines were relatively lower as compared to other ROMs. The difference found for synthetic paediatric spine and porcine spine for lateral bending was 18% while it was only 3% in axial rotation.

The average ROM in lateral bending and axial rotation of synthetic paediatric spine were within the acceptable range with porcine spine while flexion/extension differed by 45%. One of the research limitations is the simplified shape of intervertebral disc for the synthetic paediatric spine, which potentially caused a significant difference in flexion/extension. However, synthetic paediatric spine ROM exhibited a nonlinear curve for all six DOF, suggesting that the ROM measured was acceptable because the synthetic paediatric spine demonstrated a viscoelasticity behaviour that existed in human soft tissues. From the comparative analysis between the synthetic paediatric spine and porcine spine, the synthetic paediatric spine developed in this research mimicked the behaviour of biological specimen. Future works will consider using finite element analysis of paediatric spine to investigate the correct loading required in the biomechanical testing to obtain paediatric ROM.

The limitations in this study are there is no data of paediatric ROM to enable a direct comparison and the synthetic paediatric spine has to be scaled up to 200% from the actual size to fit the fixation holder in the spine simulator. Although it was a scaled-up model, the morphology of the paediatric vertebra was still maintained.

## 5. Conclusion

In the present study, fabricated synthetic paediatric spine in FSU unit was tested with a MTS Bionix Servohydraulic spine simulator to obtain the ROM in flexion, extension, lateral bending, and axial rotation. Overall, the ROM curves of synthetic paediatric spine exhibited nonlinearities as all measurements of NZ and EZ stiffness were below than 1. The ROM was then compared with the porcine spine for comparative analysis by using a comparable size model at ±4 Nm moments. The porcine spine ROM was more flexible than synthetic paediatric spine in all DOF, with a difference of 45% in flexion/extension, while the lateral bending and axial rotation of synthetic paediatric spine were in good agreement with the porcine spine, with differences of 18% and 3%, respectively. The difference in flexion/extension was potentially due to the simplified design of synthetic intervertebral disc, as it did not reflect the unique shape within the vertebral body for each individual FSU. The results presented in this research showed that the fabricated synthetic paediatric spine had nonlinearity characteristic in all DOF. The synthetic paediatric spine ROM was acceptable as compared to the porcine spine at ±4 Nm moments, specifically in lateral bending and axial rotation. Therefore, the fabricated synthetic paediatric spine particularly in thoracic region in this study can mimic the biological ROM. It could potentially be used as replacement of paediatric spine for biomechanical research that is related to spine deformity.

## Figures and Tables

**Figure 1:** Size comparison among all spine models in this study.

**Figure 2:** The process flow to manufacture paediatric synthetic spine. (a) Cortical, (b) completed vertebra, (c) disc, (d) assembled ALL and PLL, (e) added posterior ligaments, and (f) completed FSU.

**Figure 3:** The porcine specimens were dissected into single FSUs, view in (a) frontal plane and (b) transverse plane.

**Figure 4:** Experimental setup for (a) porcine spine and (b) synthetic paediatric spine in the MTS Bionix Servohydraulic spine simulator.

**Figure 5:** Typical sigmoidal curve of spine ROM.

**Figure 6:** ROM of porcine spine between this research and Wilke et al. [2] at ±7.5 Nm moments in (a) flexion extension, (b) lateral bending, (c) axial rotation, and (d) overall ROM.

**Figure 7:** Comparison between porcine spine from current study and Wilke et al. [2] with human adult spine from White and Panjabi [29].

**Figure 8:** Synthetic paediatric spine versus porcine spine at moment of ±4 Nm.

**Table 1:** Material properties of the components in the fabricated synthetic paediatric spine.

Material	Spine component	Properties		
		Compression modulus (MPa)	Tensile modulus (MPa)	Stiffness (N/mm)
Expandable polyurethane foam (0.24 g/cm^3^ density)	Trabecular bone	89.9	-	-
Urethane plastic (Smooth Cast 385)	Cortical bone	3200	-	-
Polyurethane elastomer (Monothane)	Annolous fibrosus	14.1	3.3	-
Silicone (Lightweight)	Nucleus pulposus	1.6	0.6	-
Silicone with fiber glass tape (Sorta Clear 40 in woven fibre 45°)	ALL & PLL	-	22.5	EZ = 37.8
				NZ = 109.6

**Table 2:** Porcine spine data of the ROM for each DOF of each specimen at moment of ±7.5 Nm.

FSU	ROM (°)		
	Flexion extension	Lateral bending	Axial rotation
T4-T5	6.72 ± 3.61	10.59 ± 4.87	9.51 ± 5.23
T5-T6	3.08 ± 0.19	10.46 ± 4.00	10.82 ± 4.00
T6-T7	6.69 ± 4.97	12.78 ± 8.58	16.51 ± 12.02
T7-T8	4.78 ± 1.29	12.03 ± 1.27	13.07 ± 6.95

**Table 3:** Porcine spine data of the ROM for each DOF of each specimen at moment of ±4 Nm.

FSU	ROM (°)		
	Flexion extension	Lateral bending	Axial rotation
T4-T5	1.97 ± 0.48	5.40 ± 1.00	7.15 ± 3.61
T5-T6	2.80 ± 0.28	5.60 ± 0.96	4.92 ± 0.74
T6-T7	2.47 ± 0.10	5.63 ± 1.51	7.22 ± 2.01
T7-T8	2.47 ± 0.42	6.45 ± 1.81	8.73 ± 5.80

**Table 4:** Results of the ROM and S1/S2 for each motion of synthetic paediatric specimen at moment of ±4 Nm.

FSU	Flexion extension		Lateral bending		Axial rotation	
	ROM (°)	S1/S2	ROM (°)	S1/S2	ROM (°)	S1/S2
T4-T5	0.87 ± 0.03	0.46 ± 0.28	2.46 ± 0.25	0.18 ± 0.03	3.55 ± 0.81	0.76 ± 0.05
T5-T6	0.82 ± 0.02	0.55 ± 0.09	2.89 ± 0.46	0.24 ± 0.05	3.30 ± 0.95	0.87 ± 0.04
T6-T7	1.72 ± 0.14	0.29 ± 0.16	7.00 ± 0.2	0.12 ± 0.04	9.20 ± 1.06	0.51 ± 0.25
T7-T8	1.92 ± 0.42	0.21 ± 0.06	6.56 ± 0.39	0.10 ± 0.05	11.00 ± 1.40	0.63 ± 0.15

## Data Availability

The data used to support the findings of this study are available from the corresponding author upon request.
